# Predicting Overall Survival in Patients with Nonmetastatic Gastric Signet Ring Cell Carcinoma: A Machine Learning Approach

**DOI:** 10.1155/2022/4862376

**Published:** 2022-09-13

**Authors:** Xiaomei Li, Zhiwei Chen, Jing Lin, Shouan Wang, Conghua Song

**Affiliations:** ^1^Endoscopy Center, The Affiliated Hospital (Group) of Putian University, Putian, 351100 Fujian, China; ^2^School of Basic Medicine, Medical College of Putian University, Putian, 351100 Fujian, China; ^3^Key Laboratory of Translational Tumor Medicine in Fujian Province, Putian University, Putian, 351100 Fujian, China; ^4^Department of Pathology, The Affiliated Hospital (Group) of Putian University, Putian, 351100 Fujian, China

## Abstract

**Background and Aims:**

Accurate prediction is essential for the survival of patients with nonmetastatic gastric signet ring cell carcinoma (GSRC) and medical decision-making. Current models rely on prespecified variables, limiting their performance and not being suitable for individual patients. Our study is aimed at developing a more precise model for predicting 1-, 3-, and 5-year overall survival (OS) in patients with nonmetastatic GSRC based on a machine learning approach.

**Methods:**

We selected 2127 GSRC patients diagnosed from 2004 to 2014 from the Surveillance, Epidemiology, and End Results (SEER) database and then randomly partitioned them into a training and validation cohort. We compared the performance of several machine learning-based models and finally chose the eXtreme gradient boosting (XGBoost) model as the optimal method to predict the OS in patients with nonmetastatic GSRC. The model was assessed using the receiver operating characteristic curve (ROC).

**Results:**

In the training cohort, for predicting OS rates at 1-, 3-, and 5-year, the AUCs of the XGBoost model were 0.842, 0.831, and 0.838, respectively, while in the testing cohort, the AUCs of 1-, 3-, and 5-year OS rates were 0.749, 0.823, and 0.829, respectively. Besides, the XGBoost model also performed better when compared with the American Joint Committee on Cancer (AJCC) stage. The performance for this model was stably maintained when stratified by age and ethnicity.

**Conclusion:**

The XGBoost-based model accurately predicts the 1-, 3-, and 5-year OS in patients with nonmetastatic GSRC. Machine learning is a promising way to predict the survival outcomes of tumor patients.

## 1. Introduction

Gastric cancer (GC) is the fifth most frequently diagnosed cancer worldwide and the third leading cause of cancer-related death, which has had a severe influence on global health [1, 2]. In 2020, GC caused more than 1 million new cases and approximately 770 000 deaths, with China alone accounting for approximately half (478 000) of the number of global new cases [3]. According to the WHO classification, GC can be divided into papillary adenocarcinoma, tubular adenocarcinoma, mucinous adenocarcinoma, and signet ring cell carcinoma [4]. Among them, gastric signet ring cell carcinoma (GSRC), which is named because a large amount of mucus in cancer cells pushes the nucleus to one side like a ring, is one of the most malignant tumors, accounting for about 3.4%-39% of GC [5, 6]. Though the incidence of GC has declined in the world since the active treatment of *Helicobacter pylori*, the incidence of GSRC is still increased significantly [7, 8].

GSRC is one of the types of GC with poor tissue differentiation, which has the characteristics of low differentiation, high invasiveness, and poor prognosis. Therefore, patients with GSRC often have a poorer prognosis than other types of GC [9]. According to the previous studies, GSRC is an independent factor for survival prediction, and the 5-year survival rate was 30%-46.1% [10–12]. Besides, medical decision-making in GSRC is particularly complex and requires weighing treatment benefit against tumor progression. Therefore, the development of accurate models to predict outcomes and make medical decisions is essential to improve the prognosis of patients with GSRC.

Accurate prediction is essential for the survival of patients with nonmetastatic GSRC and medical decision-making. Previous regression analysis-based models have been developed to predict the survival of patients with nonmetastatic GSRC [13–15]. Nonetheless, these models are commonly based on the assumption that each parameter, and the survival outcomes of GSRC were linear dependent (regression model). Hence, one possibility is that these models may weaken the complex relationships, which may include nonlinear associations, nonlinear interactions, or effect modification. In addition, the subjects in these studies were not followed up for more than 5 years. The model constructed based on this may have some bias in survival prediction. Therefore, there is no satisfactory survival prediction model for patients with GSRC in real-world practice [16].

To overcome this dilemma, the emerging machine learning has provided an alternative to survival prediction models. Machine learning is a data-driven application of artificial intelligence in which systems learn and improve automatically without explicit programming. It is remarkable that machine learning does not emphasize a certain assumption for data relationships but rather takes into account all possible effects between variables. Thus, machine learning is able to autonomously use datasets to identify new variables and more complex relationships between them. Its applications are rapidly growing in health care and are increasingly being used to develop novel prognostic models for several diseases [17]. Besides, using machine learning methods to construct prediction models for the survival of cancer patients has been proven to be more accurate, robust, and generalizable [17–19].

Our study is aimed at developing a more precise model for predicting 1-, 3-, and 5-year overall survival (OS) in patients with nonmetastatic GSRC based on machine learning approaches. Instead of single information derived from image segmentation or image recognition based on artificial intelligence, the parameters used in machine learning for modeling here were the more dimensional data derived from clinical practice. The significance of this study not only lies in the development of prediction model for GSRC survival but also includes a call for action to reduce the bias of survival prediction studies in the field of gastrointestinal tumors.

## 2. Methods

### 2.1. Data Source and Study Population

The data was collected from the Surveillance, Epidemiology, and End Results (SEER) program with the National Cancer Institute's SEER∗Stat software (version 8.3.9, http://seer.cancer.gov/seerstat/). SEER collects cancer diagnoses and survival data for approximately 30% of the US population and benefits from extensive quality review model development. GSRC patients were preliminarily screened according to the International Classification of Diseases in Oncology (ICD-O-3) and histology code (8490/3).

Patients were further screened according to the following criteria: the inclusion criteria were (1) patients diagnosed in 2004−2014, (2) ICD-O-3 identified the primary site as the stomach, (3) patients with only one primary tumor, and (4) patients with complete survival information. The exclusion criteria were (1) patients with distant metastasis of tumor, (2) tumor grade or race or tumor size unknown, (3) TNM or the American Joint Committee on Cancer (AJCC) stage unknown, (4) surgical information unknown, and (5) age less than 15 or more than 90 years old.

We collected the following variables from the SEER database: age, sex, race, marital status, tumor location, tumor size, histologic grade, T stage, N stage, number of regional lymph nodes (LNs) examined, AJCC stage, and survival month. Finally, a total of 2127 patients were included in our study and then randomly assigned with R 3.6.1 to the training cohort and the validation cohort at a ratio of 7 to 3. Access to the SEER database does not require formal ethical approval, and its open access policy is included. The detailed screening process for GSRC patients is shown in Figure 1.

### 2.2. Study Design

Race was classified into three types: White, Black, and other. Marital status was recorded as married and unmarried. The grade was classified into four types: well-differentiated (grade I), moderately differentiated (grade II), poorly differentiated (grade III), and undifferentiated/anaplastic (grade IV). Historic stage A was recorded as localized, regional, or distant. T stage was recorded as T1, T2, T3, or T4. N stage was recorded as N0 (negative), N1 (1-2 positive LNs), N2 (3-6 positive LNs), or N3 (>6 positive LNs).

Previous studies classified the number of examined LNs into two types: regional nodes examined ≤16, and regional nodes examined >16 [19]. All patients were restaged according to AJCC criteria described in AJCC 8^th^ edition staging manual [20] and recorded as I, II, III, and IV. Tumor size was categorized into 6 groups: ≤1 cm, 1-2 cm, 2-3 cm, 3-4 cm, 4-5 cm, and >5 cm. The primary sites were recorded as the cardia, fundus, body, antrum, pylorus, lesser curvature, greater curvature, and overlapping lesion/not otherwise specified (NOS). The therapy was recorded as none, surgery only, chemo/radio only, and surgery plus chemo/radio. The primary outcome was the prediction of OS rate at 1-, 3-, and 5-year, assessed in patients aged 15–90 years with nonmetastatic GSRC.

### 2.3. Model Development

To improve the accuracy of our model, the following variables were included: age, sex, race, marital status, tumor location, tumor size, histologic grade, T stage, N stage, and the number of regional LNs examined. The training cohort was used to train an eXtreme gradient boosting model (with the XGBoost package in R), and the validation cohort was used to verify the model's accuracy.

Before choosing and optimizing the XGBoost model, we performed rigorous exploratory analyses of k-nearest neighbor (KNN), support vector machines (SVM), random forest (RF), and neural networks (NT). Separate models were generated with hyperparameter tuning to optimize their performance for each outcome, and all models underwent validation using the validation cohort. The receiver operating characteristic curve (ROC), the area under ROC (AUC), and the accuracy were used to assess the precision and specificity of models. The AUC ranges from 0 to 1, with 1 indicating perfect concordance, 0.5 indicating no better concordance than chance.

The preliminary findings suggested that RF and XGBoost appeared to perform better than other models in the training cohort (Table 1). However, in the validation group, the performance of the RF algorithm is poor, which means that the RF algorithm may have an overfitting phenomenon. Hence, we chose the XGBoost algorithm as our final model. XGBoost is a regression tree algorithm based on machine learning, which combines the outputs of other decision trees to improve the classification. XGBoost is a recently developed gradient tree boosting algorithm, which is scalable and allows faster calculations [21].

### 2.4. Statistical Analysis

All analyses were performed using R statistical software 3.6.1 (http://www.r-project.org). For normally distributed data, continuous variables were expressed as mean ± standard deviation (SD). Categorical variables were presented as proportions. Variables with *P* < 0.05 were taken into consideration as significant.

## 3. Results

### 3.1. Baseline Characteristics of Patients

Figure 1 shows our data assembly process. Between 2004 and 2014, a total of 7124 patients from the SEER database with histologically confirmed GSRC were enrolled in our study. Of these, 3562 patients who presented with evidence of distant metastasis were excluded. 1198 patients had missing data for tumor grade or race or tumor size, 215 patients did not have TNM or AJCC stage information, 3 patients did not have surgical information, and 19 people outside of the study age range (15–90 years) were also excluded.

The final study population included 2127 patients. Baseline characteristics of the study cohort were shown in Table 2. The mean age was 61.6 ± 0.31 years old. 1100 (51.7%) were male. Most patients were White (65.5%), and 15% were Black. 60.4% of patients were married. The primary grade was grade III (93.7%), the central stage A was regional (63.1%), and the main AJCC stage was I (32.3%). Meanwhile, 930 patients (43.7%) had a tumor size >5 cm. T1 (41.9%), N0 (35.4%), and regional nodes examined ≤16 (56%) accounted for predominance. The gastric antrum was the most common site for GSRC (25.5%). Among all included patients, the OS rates at 1, 3, and 5 years were 72.4%, 42.1%, and 29.4%, respectively.

### 3.2. Performance of the ML Model

Figure 2 shows the ROC of different machine learning models in predicting the OS of GSRC. Table 1 shows the AUC with 95% CI of different machine learning models in predicting the OS of GSRC. We can see that the XGBoost model performed well both in the training and testing cohorts. In the training cohort, for predicting OS rate at 1, 3, and 5 years, the AUCs of the XGBoost model were 0.842, 0.831, and 0.838, respectively, while in the testing cohort, the AUCs of 1-, 3- and 5-year OS rates were 0.749, 0.823, and 0.829, respectively.

Next, we established the ROC curve and calculated the corresponding AUC to compare the XGBoost model and AJCC staging accuracy in predicting patients' OS. As shown in Figure 3, the 1-, 3-, and 5-year AUCs predicted by ROC analysis of the XGBoost model were significantly higher than the AUC values calculated from the AJCC staging system. It means that the XGBoost model had superior predictive ability to the AJCC staging system. Besides, we also compared the 1-, 3-, and 5-year AUCs of the XGBoost model stratified by age and race.

In our study, model performance was marginally better in men aged 65 years or older than in men younger than 65 (Table 3 and Figure 4). And the model was the best in predicting the 5-year OS rate of people aged 65 years or older (AUC: 0.849, 95% CI: 0.820-0.878). Then, we tested performance in different ethnic groups. The XGBoost model also performed well (Table 4 and Figure 5). The significance of the predictors in the XGBoost model is presented in Figure 6. The most important predictor was the T stage, followed by age, therapy, primary site, and tumor size.

## 4. Discussion

GSRC is a highly malignant type of GC, accounting for 8-30% of GC cases [22, 23]. Although the incidence rates of GSRC are low, its reported 5-year survival rate was only 15.9% [24]. Besides, the prognosis of GSRC remains controversial. Previous studies demonstrated that the survival of GSRC patients was relatively better than other histological types in the early stage. Probably because the tumor of GSRC is more frequently found in early-stage GC, the early-stage GSRC has a lower risk of lymph node metastasis [12, 25–27]. However, study about the accurate prognosis of early GSRC is rare. Hence, it is imperative to establish a predictive model to guide the clinical work better.

In this study, we used a large and public dataset to construct and validate a machine learning-trained prognostic model for predicting 1-, 3-, and 5-year OS rates in patients with nonmetastatic GSRC and assessed its performance against the eighth edition AJCC staging system. To our best knowledge, our study is the first to use the SEER cohort to establish a machine learning model for predicting OS rate in patients with nonmetastatic GSRC.

AJCC staging system currently used prognostic GC patients. However, the current GC monitoring prediction model is not suitable for the tracking of GSRC. Notably, the AJCC staging system does not account for some significant clinicopathological characteristics, such as age, gender, and treatment method, which were all related to patients' survival. In the present study, our model incorporated the above characteristics into machine learning, and the results showed our model's performance was better than the AJCC staging system.

Prior research has been carried out to develop simple multivariable regression predictive models for GSRC. Xu et al. developed a prognostic nomogram based on log odds of positive lymph nodes to predict the OS and CSS rate of GSRC [12]. However, the model was not good at predicting the 1-year OS rate (AUC: 0.768), and its 5-year OS rate prediction ability showed only a slight preponderance over AJCC. Besides, this study selected patients diagnosed from 2010 to 2015 from the SEER database, and the database only has follow-up data up to 2018. Hence, there may be a certain deviation for this study in predicting the 5-year OS rate.

The studies carried out by Wang et al., Zhang et al., and Guo et al. also had similar problems [13, 14, 28]. Wei et al. collected 1,030 patients from the SEER database and constructed CSS prognostic model. They found that patients who received postoperative radiotherapy had a better prognosis than patients who underwent surgery alone [29]. Guo et al. constructed a nomogram predicting lymph node metastasis [30]. However, these studies have limited population selection, and the predictive ability is not good.

Many consider machine learning as a “black box,” in which a computer generates predictions. Unfortunately, most clinicians have a limited understanding of the machinations involved to generate these predictions. While medicine remains behind other disciplines in utilizing machine learning, its predictive power has been demonstrated with increasing frequency [16, 17, 31, 32]. Compared with the traditional parametric model, machine learning has more flexible, accurate, and robust predictive capabilities [17]. Besides, machine learning methods based on specific samples with explicit characteristic attributes are more suitable for identifying individual patients [33].

In recent years, the research on medical image diagnosis based on artificial intelligence has increased significantly. Different image vision classification and image segmentation tools can be used to identify abnormalities caused by diseases. Compared with manpower, the main advantages of image information capture technology based on artificial intelligence are fast detection speed, high accuracy, and stable results. However, instead of single information derived from image segmentation or image recognition based on artificial intelligence, the parameters used in machine learning for modeling here were more dimensional data from clinical practice. XGBoost is a regression tree algorithm based on machine learning, which combines the outputs of other decision trees to improve the classification and allows faster calculations.

XGBoost, a regression tree algorithm for faster calculations, is recently developed as an open source project. The whole execution process of XGBoost is easy and can run as packages in a freely available language R 3.6.1. In our study, by comparing several other algorithms, we chose the XGBoost algorithm for modeling. XGBoost algorithm has the advantages of regularization and parallel processing, which made the model perform well in our research [34].

Although our model has a satisfactory accuracy, several limitations also deserve to be mentioned. First, though SEER is a huge population-based database, some critical information was not explained, potentially making the models even more accurate. Second, the model was constructed using a retrospective nationwide database. Therefore, the current analysis of the patient population could not exclude the possibility of selection bias. Finally, external validation is lacking in this study. Further study is needed to validate the advantages of the model in survival prediction.

In conclusion, this study is the first to explore the performance of machine learning in predicting OS in patients with nonmetastatic GSRC. XGBoost is a regression tree algorithm based on machine learning, which combines the outputs of other decision trees to improve the classification and allows faster calculations. The XGBoost-based model accurately predicts the 1-, 3-, and 5-year OS in patients with nonmetastatic GSRC. Machine learning is a promising way to predict the survival outcomes of tumor patients.

## Figures and Tables

**Figure 1:** The flowchart of patients included in the present study.

**Figure 2:** A comparison of the area under the receiver operating characteristic curve (AUROC) of different machine learning models in predicting (a) 1-, (b) 3-, and (c) 5-year overall survival (OS) in patients with nonmetastatic GSRC in the training cohort and (d) 1-, (e) 3-, and (f) 5-year OS in the validation cohort. KNN: k-nearest neighbor; SVM: support vector machines; RF: random forest; NT: neural networks; XGB: an eXtreme gradient boosting.

**Figure 3:** A comparison of the area under the receiver operating characteristic curve (AUROC) of eXtreme gradient boosting (XGB) and the American Joint Committee on Cancer (AJCC) stage in predicting (a) 1-, (b) 3-, and (c) 5-year overall survival (OS) in the training cohort and (d) 1-, (e) 3-, and (f) 5-year OS in the validation cohort.

**Figure 4:** The area under the receiver operating characteristic curve (AUROC) of the eXtreme gradient boosting model in predicting (a) 1-, (b) 3-, and (c) 5-year overall survival (OS) in patients aged < 65 years old and (d) 1-, (e) 3-, and (f) 5-year OS in patients age ≥ 65 years old.

**Figure 5:** The area under the receiver operating characteristic curve (AUROC) of the eXtreme gradient boosting model in predicting (a) 1-, (b) 3-, and (c) 5-year overall survival (OS) in the White race; (d) 1-, (e) 3-, and (f) 5-year OS in the Black race; and (g) 1-, (h) 3-, and (i) 5-year OS in the other race.

**Figure 6:** Significance of the predictors in the eXtreme gradient boosting model.

**Table 1:** Performance of machine learning models in OS.

Model	Training cohort	Testing cohort
	AUC with 95% CI	AUC with 95% CI
1-year survival		
KNN	0.773 (0.747-0.799)	0.715 (0.669-0.760)
Support vector machines	0.784 (0.757-0.810)	0.738 (0.695-0.782)
Random forest	0.998 (0.997-0.999)	0.725 (0.681-0.770)
XGBoost	0.842 (0.819-0.863)	0.749 (0.708-0.791)
Neural network	0.789 (0.764-0.815)	0.706 (0.662-0.751)
3-year survival		
KNN	0.801 (0.779-0.823)	0.800 (0.766-0.835)
Support vector machines	0.795 (0.773-0.818)	0.812 (0.779-0.846)
Random forest	0.997 (0.995-0.998)	0.807 (0.773-0.841)
XGBoost	0.831 (0.811-0.852)	0.823 (0.790-0.854)
Neural network	0.814 (0.792-0.836)	0.765 (0.729-0.802)
5-year survival		
KNN	0.813 (0.791-0.836)	0.765 (0.725-0.806)
Support vector machines	0.813 (0.789-0.836)	0.774 (0.733-0.815)
Random forest	0.996 (0.994-0.998)	0.774 (0.734-0.814)
XGBoost	0.838 (0.816-0.858)	0.829 (0.793-0.863)
Neural network	0.811 (0.787-0.836)	0.776 (0.737-0.815)

**Table 2:** Demographic and clinicopathological characteristics of patients.

Variables	All patients (*n* = 2127)	Training cohort (*n* = 1488)	Validation cohort (*n* = 639)
Age (year, mean ± SD)	61.6 ± 0.31	61.37 ± 0.37	62.15 ± 0.55
Sex (no. (%))			
Female	1027 (48.3)	701 (47.1)	326 (51)
Male	1100 (51.7)	787 (52.9)	313 (49)
Race (no. (%))			
White	1393 (65.5)	975 (65.5)	418 (65.4)
Black	318 (15)	215 (14.4)	103 (16.1)
Other	416 (19.5)	298 (20)	118 (18.5)
Marital status (no. (%))			
Married	1284 (60.4)	909 (61.1)	375 (58.7)
Unmarried	843 (39.6)	579 (38.9)	264 (41.3)
Grade (no. (%))			
I	3 (0.1)	1 (0.1)	2 (0.3)
II	63 (3)	46 (3.1)	17 (2.7)
III	1992 (93.7)	1392 (93.5)	600 (93.9)
IV	69 (3.2)	49 (3.3)	20 (3.1)
Size (no. (%))			
≤1 cm	128 (6)	90 (6)	38 (5.9)
1-2 cm	278 (13.1)	187 (12.6)	91 (14.2)
2-3 cm	315 (14.8)	220 (14.8)	95 (14.9)
3-4 cm	258 (12.1)	191 (12.8)	67 (10.5)
4-5 cm	218 (10.2)	149 (10)	69 (10.8)
>5 cm	930 (43.7)	651 (43.8)	279 (43.7)
Stage A (no. (%))			
Localized	652 (30.7)	460 (30.9)	192 (30)
Regional	1343 (63.1)	935 (62.8)	408 (63.8)
Distant	132 (6.2)	93 (6.3)	39 (6.1)
T stage (no. (%))			
T1	428 (20.1)	296 (19.9)	132 (20.7)
T2	892 (41.9)	637 (42.8)	255 (39.9)
T3	609 (28.6)	417 (28)	192 (30)
T4	198 (9.3)	138 (9.3)	60 (9.4)
N stage (no. (%))			
N0	754 (35.4)	530 (35.6)	224 (35.1)
N1	739 (34.7)	504 (33.9)	235 (36.8)
N2	424 (19.9)	299 (20.1)	125 (19.6)
N3	210 (9.9)	155 (10.4)	55 (8.6)
Site (no. (%))			
Cardia	351 (16.5)	259 (17.4)	92 (14.4)
Fundus of stomach	67 (3.1)	44 (3)	23 (3.6)
Body of stomach	220 (10.3)	162 (10.9)	58 (9.1)
Gastric antrum	543 (25.5)	375 (25.2)	168 (26.3)
Pylorus	185 (8.7)	131 (8.8)	54 (8.5)
Lesser curvature of stomach	111 (5.2)	82 (5.5)	29 (4.5)
Greater curvature of stomach	271 (12.7)	189 (12.7)	82 (12.8)
Overlapping/NOS	379 (17.8)	246 (16.5)	133 (20.8)
Therapy (no. (%))			
None	61 (2.9)	39 (2.6)	22 (3.4)
Surgery only	728 (34.2)	511 (34.4)	217 (34)
Chemo/radio only	158 (7.4)	113 (7.6)	45 (7)
Surgery plus chemo/radio	1180 (55.5)	825 (55.4)	355 (55.6)
Regional nodes examined (no. (%))			
≤16	1192 (56)	825 (55.4)	367 (57.4)
>16	935 (44)	663 (44.6)	272 (42.6)
AJCC (no. (%))			
I	686 (32.3)	476 (32)	210 (32.9)
II	473 (22.2)	325 (21.8)	148 (23.2)
III	637 (29.9)	450 (30.2)	187 (29.3)
IV	331 (15.6)	237 (15.9)	94 (14.7)
Overall survival (no. (%))			
1 years	1540 (72.4)	1080 (72.6)	460 (72)
3 years	895 (42.1)	623 (41.9)	272 (42.6)
5 years	625 (29.4)	440 (29.7)	185 (29)

**Table 3:** Performance of XGBoost models in OS stratified by age.

	Age < 65 years^∗^	Age ≥ 65 years^∗^
1-year survival	0.710 (0.677-0.744)	0.749 (0.718-0.781)
3-year survival	0.796 (0.771-0.822)	0.832 (0.804-0.859)
5-year survival	0.805 (0.779-0.832)	0.849 (0.820-0.878)

^∗^AUC with 95% CI.

**Table 4:** Performance of XGBoost models in OS stratified by race.

	White^∗^	Black^∗^	Other^∗^
1-year survival	0.744 (0.716-0.771)	0.729 (0.666-0.792)	0.755 (0.699-0.810)
3-year survival	0.816 (0.794-0.839)	0.788 (0.737-0.838)	0.849 (0.812-0.885)
5-year survival	0.817 (0.793-0.842)	0.848 (0.800-0.896)	0.840 (0.801-0.878)

^∗^AUC with 95% CI.

## Data Availability

Available datasets were analyzed in this study. This data can be found in https://seer.cancer.gov/data/. Further enquiries can be directed to the corresponding author.

## Abbreviations

GSRC: Gastric signet ring cell carcinoma
OS: Overall survival
SEER: Surveillance, Epidemiology, and End Results
ROC: Receiver operating characteristic curve
XGBoost: eXtreme gradient boosting
AJCC: American Joint Committee on Cancer
GC: Gastric cancer
ICD: International Classification of Diseases
LN: Lymph node
KNN: K-nearest neighbor
SVM: Support vector machines
RF: Random forest
NT: Neural networks.
